# Improved glycemic status, insulin resistance and inflammation after receiving oral oleoylethanolamide supplement in people with prediabetes: a randomized controlled trial

**DOI:** 10.1186/s13098-022-00848-3

**Published:** 2022-06-03

**Authors:** Elahe Pouryousefi, Maryam Javadi, Sima Hashemipour, Mohamadreza Rashidi Nooshabadi, Hossein Khadem Haghighian

**Affiliations:** 1 Department of Nutrition, School of Health, Qazvin University of Medical Sciences, Qazvin, Iran; 2 Children Growth Research Center, Research Institute for Prevention of Non-Communicable Diseases, Qazvin University of Medical Sciences, Qazvin, Iran; 3 Metabolic Diseases Research Center, Research Institute for Prevention of Non-Communicable Diseases, Qazvin University of Medical Sciences, Qazvin, Iran; 4 Department of Pharmacology, School of Pharmacy, Ahvaz Jundishapur University of Medical Sciences, Ahvaz, Iran; 5 Department of Nutrition, School of Health, Qazvin University of Medical Sciences, Qazvin, Iran

**Keywords:** Oleoylethanolamide, Glycemic status, Insulin resistance, Prediabetes

## Abstract

**Background:**

The anti-inflammatory properties of cannabinoids have been shown. This study was conducted to assess effect of oleoylethanolamide (OEA) supplementation on glycemic status, insulin resistance (IR) and inflammatory factor in pre-diabetic individuals.

**Methods:**

This double-blind randomized clinical trial was done at Qazvin University of Medical Sciences in which 46 pre-diabetic patients were divided into two equal groups and received one 125 mg OEA capsule in the intervention group (23 subjects) and 125 mg capsule containing wheat flour in placebo group daily for 8 weeks. After collecting demographic information, at the beginning and end of the study, the questionnaires of physical activity, 24-hour food recall were completed and blood glucose (BG), plasma insulin level, IR, hemoglobin A_1_c (HbA_1_c), and C-reactive protein (CRP) were measured. Statistical analysis was performed using SPSS software.

**Results:**

At the beginning and end of the study, there was no significant difference between the two groups in terms of anthropometric indices, food intake and physical activity (P > 0.05). At the end of the study, consumption of OEA significantly reduced BS, insulin, IR, HbA_1_c, and CRP (P < 0.05). No significant change was observed in mentioned biochemical factors in placebo group (P > 0.05).

**Conclusions:**

Given that OEA supplementation improved the glycemic status, IR and reduced the inflammatory factor, use of this supplement can be introduced as a useful supplement to control pre-diabetes status.

*Trial registration*: The protocol of this clinical trial is registered with the Iranian Registry of Clinical Trials (http://www.IRCT.IR, identifier: IRCT20141025019669N16).

## Background

Prediabetes is a metabolic condition that is the boundary between healthy people and people with diabetes. Prediabetes is a condition in which people have impaired fasting glucose(IFG) [1]. In these people, fasting blood glucose (FBG) is between 100 and 125 mg/dL and also 2 h after consuming 75 g of oral glucose is 140–199 mg/dL or the amount of glycosylated hemoglobin (HbA_1_C) is 5.7–6.4%. According to studies, the rate of impaired glucose tolerance in 2019 is 373.9 million people which is predicted to reach 548.4 million by 2045 [2]. A condition that worsens the pathophysiological condition of people with pre-diabetes is the development of insulin resistance (IR) in their body. The cells’ resistance to insulin and the inability of the receptors to work with this hormone disrupt the function of pancreatic beta cells, which is usually seen before diabetes. Continuation of this condition and increase IR, can lead to high blood glucose, which can lead to increased inflammation and oxidative stress (OS). These long-term complications can lead to microangiopathy and cardiovascular disease [3]. In a study in 2019, it was found that IR was associated with OS in non-diabetic people. This connection becomes stronger, especially in people who are overweight or have impaired fasting glucose tolerance [4]. The results of a study by Sthijns et al., in 2020 showed that increasing reactive oxygen species (ROS) and stabilizing OS could lead to impaired glucose uptake by muscle and adipose tissue and reduced insulin secretion from beta cells [5]. Many drugs are used to control and treat prediabetes, such as Biguanides, sulfonylureas, alpha glucosidase inhibitors and GLP1 analogues [6]. Although according to recent studies, metformin is mainly used to control and treat pre-diabetes along with healthy diet and increased physical activity, but the results of clinical studies show that lifestyle interventions causes better control of these conditions and also effective in reducing the conversion of prediabetes to diabetes [7]. Reducing calorie intake in prediabetic people for weight loss is one of the basic recommendations and moderate to vigorous physical activity of 150 min per week is effective in preventing diabetes, especially when it is a combination of aerobic and strength training [8]. Recent studies show that prediabetes can lead to changes in inflammatory cytokines. One of the causes of inflammation is the accumulation of triglycerides in non-adipose tissues. Cannabinoids are active compounds derived from lipids [9]. There are several roles for cannabinoids, such as weight loss, appetite control, and inflammation control [10]. Some studies have shown anti-inflammatory, antioxidant and antidiabetic properties for cannabinoids [11]. One of the endocannabinoids compounds is oleoylethanolamide (OEA), a small amount of which is naturally occurring in the intestinal tract. OEA has several roles, including improving the inflammatory process, boosting the immune system, stimulating lipolysis, and lipid oxidation. This fatty acid belongs to the N-acetyl ethanolamides family, which is derived from the monounsaturated fatty acid oleic acid [12]. In some studies, OEA has been linked to decreased appetite and control of inflammation [13]. In a review study, Tutunchi et al. Showed that administering or receiving OEA could be effective in reducing inflammation [14]. Due to the importance of the inflammatory process in the progression of diabetes and the observed effects of OEA on reducing the inflammatory process and risk of diabetes, the present study is dedicated to this topic. The aim of this study was to evaluate the effect of OEA supplementation on glycemic status, IR and inflammatory factor in pre-diabetic individuals.

## Material and method

### Ethics

This scientific project was approved by the ethics code of IR.QUMS.REC.1399.482 in the ethics committee of the research deputy of Qazvin University of Medical Sciences and was registered with the identification code of IRCT20141025019669N16 in clinical trials registry of Iran. In this scientific study, all participants signed written consent with full awareness about this clinical program.

### Inclusion and exclusion criteria

At the beginning of study, 52 pre-diabetic patients who referred to the endocrinology and metabolism clinic of Qazvin University of Medical Sciences, Qazvin, Iran in 2020 and approved by a specialist were included in the study. According to the American Diabetes Association (ADA), pre-diabetes is a condition that the patient has impaired fasting glucose tolerance (IFG; 100 mg/dL to 125 mg/ dL) and/or impaired glucose tolerance (IGT; 2 h plasma glucose in the 75 gr; oral glucose tolerance test (OGTT) 140 mg/dL to 199 mg/dL) and/or HbA1c 5.7–6.4 [15].

### Patients

Individuals with the mentioned inclusion criteria as well as willing to cooperate and with moderate level of physical activity were included in the study. Pregnancy and lactation, Body mass index (BMI) > 30, severe renal and hepatic impairment, change in dose of antihypertensive drugs, change in diet, change in physical activity, taking any dietary supplement from 2 months ago, unwillingness to participate in the study, history of any allergies and alcohol consumption were the exclusion criteria.

### Study design

This randomized controlled trial had two parallel groups and was randomly blinded with a control group that designed to evaluate the effect of the OEA supplementation on some laboratory factors in prediabetes patients. Patients were divided into two groups OEA (n = 23) and placebo (n = 23) randomly using random numbers. The intervention group received 125 mg of OEA daily and the placebo group received similar capsule containing wheat flour for two months. In this double-blind study, factors that could distort the test result, such as information about supplementation or placebo, were hidden from both the participant (patients) and the researcher. The effective dose for supplementation of OEA was taken from the article of Payahoo L et al. [16]. The supplement was bought from a SupplementSpot and the placebo was made by School of Pharmacy, Tabriz University of Medical Sciences. The color, shape, and size of the supplement capsules were similar to those of the placebo capsules. Patients were told to take the capsules with the main meal. Questionnaires including personal information and medical records were filled out by the trainee. It should be noted that all participants in this project were taking metformin. In order to control the confounding factors in the clinical study such as diet and physical activity, questionnaires related to the physical activity level and food recall (3-day non-consecutive food recall questionnaire, 2 normal days and one day off) were completed through interviews. Patients were advised by researchers to avoid dietary changes and physical activity during the study to control confounding factors. Analysis of food recall questionnaires was performed using Nutritionist IV program (San Bruno, CA) modified for Iranian food composition. Physical activity was measured at the beginning and end of the eighth week by completing a valid and reliable questionnaire (International Questionnaire Activity Physical (IPAQ) [17] through interviews with individuals. Daily telephone follow-up was performed to check the use of supplements. At the end of the intervention, patients referred to the laboratory for blood sampling and questionnaires related to the control of confounders were completed at the end of the study.

### Biochemical measurements

At the beginning and end of the study, 10 cc of venous blood samples were taken and after separation of serum, biochemical parameters of glycemic status including fasting blood glucose (FBG), 2-hour Post Prandial (2hpp), (2-hour after breakfast), and HbA1c%, insulin and CRP measured in the plasma of the participants. Tubes with and without EDTA were used to collect blood samples. Tubes without EDTA were centrifuged (Beckman Avanti J-25, USA, 3000 rpm,10 min) and finally maintained at minus − 70 ° C for final measurements. FBG concentration was measured by the enzymatic method using an Abbot ModelAclyon 300, USA auto analyzer with Pars-Azmone kit (Tehran, Iran). The percentage of HbA1c was determined by high performance liquid chromatography (HPLC). Plasma insulin was measured by using a chemiluminescent immunoassay method (LIAISON analyzer (310,360) Diasorin S.P.A., Verecelli, Italy). Insulin resistance (IR) was calculated according to the following formula: Homeostatic Model Assessment for Insulin Resistance (HOMA-IR) (µU/ml) = (Fasting insulin (U/ml) × FBG (mg/dl)/405) [18]. CRP concentration was measured by using an immune turbid metric assay (Pars Azmoon kit. Iran).

### Sample size

FBG values before and after OEA administration were used in the study of Tutunchi H et al. [19], using the following formula to calculate the sample size.

$${\text{N}} = {\text{ }}\left[ {\left( {{\text{Z}}_{{{\text{1}} - \alpha /{\text{2}}}}  + {\text{ Z}}_{{{\text{1}} - \beta }} } \right)^{{\text{2}}} \left( {{\text{SD}}_{{\text{1}}} ^{{\text{2}}}  + {\text{SD}}_{{\text{2}}} ^{{\text{2}}} } \right)} \right]{\text{ }}/\Delta ^{{\text{2}}}$$

Where a (type 1 error) is 0.05, b (type 2 error) is 0.2, SD and ∆ the variances and difference means of FBG, respectively. Thus, the power for detecting differences between the 2 groups for various outcomes in the present study was 80%. The sample size was obtained 15 in each group. Considering probable drop-out, the sample size was considered 22. In this research, 44 pre-diabetic patients were studied.

### Statistical analyses

Statistical analyses were conducted using SPSS version 20. All data were presented as mean ± SD and were checked for normality by the Kolmogorov–Smirnov test. Due to the normal distribution of variables, the paired sample t-test and the independent sample t-test were applied to analyze differences in variables within and between groups, respectively. The p < 0.05 was considered statistically significant. To control confounding variables, analysis of covariance (ANCOVA) test were used to determine the differences between the two groups post-intervention, while adjusting for baseline measurements and covariates. Differences were considered statistically significant at P < 0.05. In this study, Intention-to-treat analysis was not used.

## Results

In this study, 46 pre-diabetic patients participated who were randomly assigned to one of the intervention groups (23 patients) and the placebo group (23 patients). During this study, three patients (one patient in the intervention group and two patient in the placebo group) could not continue the study due to personal reasons and were excluded from the study whose data were excluded from the final statistical analysis (Fig. 1). The participation rate of the participants in this study was 93.47%. The flow chart of the selected participants is shown in Fig. 1. Also, no side effects from supplementation or placebo were reported in this study.

**Fig. 1:** Trial profile and design

Information about the participants is shown in Table 1. There was no statistically significant difference in the basic characteristics of the participants between the two groups. The mean age of participants in the intervention and placebo groups was 49.64 ± 7.932 and 49.76 ± 8.105 years, respectively. At the beginning of the study, there was no significant difference between the two groups in terms of weight, body mass index, physical activity, metformin dose and duration of diabetes. Also, the average energy intake, macronutrients and some micronutrients at the beginning and end of the study are given in Table 2. As it turns out, there was no significant difference in daily energy intake, macronutrients and some other nutrients. Also, at the end of the study, the amount of changes in these factors compared to the first study was not statistically significant (Table 2).

**Table 1:** The comparison of baseline characteristics of the participants

Variable	Mean ± SD Placebo (n = 21)	Mean ± SD Oleoylethanolamide (n = 22)	P1
Age (years)	49.76 ± 8.10	49.64 ± 7.93	0.529
Height (cm)	163.71 ± 9.12	162.43 ± 10.59	0.614
Weight (kg)			
Before	73.55 ± 8.99	71.83 ± 7.89	0.512
After	72.63 ± 10.37	70.49 ± 11.33	0.419
P2	0.58	0.61	
Body mass index (K g/m²)			
Before	27.44 ± 1.9	27.22 ± 1.07	0.329
After	27.09 ± 1.26	26.71 ± 1.1	0.307
P2	0.3	0.291	
Physical activity (met-h/week)			
Before	38.19 ± 5.48	39.02 ± 8.25	0.39
After	39.06 ± 6.11	40.66 ± 9.11	0.402
P2	0.404	0.41	
Metformin dose (mg)	1023 ± 206.07	1040.25 ± 219.17	0.63

Data are expressed as means ± SD

P1: Mean comparison of the baseline characteristics between the two groups of OEA and placebo (Independent samples t-test)

P2: Mean comparison of the baseline characteristics in each group at baseline and end of study (Paired samples t-test)

**Table 2:** The comparison of the dietary intake at the baseline and the end of the study in participants

Variables	Mean ± SD Placebo (n = 21)	Mean ± SD Oleoylethanolamide (n = 22)	P1
Energy (kcal)			
Baseline	2224.14 ± 398.017	2173.6 ± 357.01	0.704
End	2197.81 ± 401.19	2133.05 ± 390.44	0.652
P2	0.691	0.709	
Protein (gr)			
Baseline	75.03 ± 23.17	73.26 ± 20.53	0.26
End	73.11 ± 25.14	71.03 ± 22.33	0.2
P2	0.29	0.24	
Carbohydrate (gr)			
Baseline	290.93 ± 85.29	286.45 ± 90.17	0.551
End	285.52 ± 63.11	280.22 ± 74.36	0.509
P2	0.521	0.303	
Fat (gr)			
Baseline	83.07 ± 19.31	81.19 ± 17.44	0.22
End	80.64 ± 18.65	78.24 ± 15.59	0.198
P2	0.209	0.21	
Saturated fatty acids (gr)			
Baseline	29.08 ± 10.31	28.57 ± 9.23	0.11
End	27.1 ± 9.07	26.06 ± 8.37	0.104
P2	0.107	0.1	
Monounsaturated fatty acid (gr)			
Baseline	25.11 ± 6.5	23.55 ± 4.13	0.091
End	25.17 ± 6.19	22.14 ± 5.09	0.1
P2	0.19	0.1	
Polyunsaturated fatty acid (gr)			
Baseline	26.77 ± 8.06	25.19 ± 9.11	0.12
End	25.39 ± 7.85	24.66 ± 9.03	0.091
P2	0.11	0.1	
Fiber (gr)			
Baseline	12.36 ± 4.14	12.01 ± 2.17	0.079
End	11.52 ± 3.28	11.6 ± 3.39	0.072
P2	0.071	0.074	
Vitamin C (mg)			
Baseline	73.06 ± 21.36	70.65 ± 19.28	0.31
End	70.44 ± 20.99	71.25 ± 23.14	0.33
P2	0.301	0.39	
Vitamin E (IU)			
Baseline	12.23 ± 4.55	11.44 ± 3.81	0.061
End	12.09 ± 3.61	10.33 ± 3.19	0.058
P2	0.066	0.06	
Selenium (µgr)			
Baseline	125.03 ± 39.14	123.75 ± 42.66	0.3
End	123.11 ± 41.18	122.96 ± 39.04	0.32
P2	0.29	0.32	

Data are expressed as means ± SD

P1: Mean comparison of the baseline characteristics between the two groups of OEA and placebo (Independent samples t-test)

P2: Mean comparison of the dietary intake in each group at baseline and end of study (Paired samples t-test)

The effect of OEA supplementation on glycemic status, insulin resistance and CRP in participants is summarized in Table 3. The data in the table indicate that, at the beginning of the study, there was no significant difference between these factors (P > 0.05). At the end of the study, supplementation significantly reduced the mean FBG, 2-hp, and HbA1c (%), insulin and HOMA-IR in the intervention group compared with the placebo group (P < 0.05). Also, intra-group comparison showed that at the end of the study in the intervention group, there is a statistically significant difference compared to the beginning of the study (P < 0.05). However, the mean changes at the end of the study were not statistically significant in the placebo group compared to the first study (P > 0.05). The mean HOMA-IR index before the intervention was not significantly different between the two groups, but after the intervention there was a significant difference between the two groups (P < 0.05). Also, supplementation with OEA caused a statistically significant decrease in the mean of CRP in the intervention group compared with the placebo group (P < 0.05). Also, changes within the group showed that there was a statistically significant difference compared to the beginning of the study in the intervention group. However, the mean changes between the beginning and end of the study in the placebo group were not statistically significant (P > 0.05, Table 3).

**Table 3:** Changes in baseline to endpoint measures for glycemic status and inflammatory factor in two groups

Variables	Mean ± SD Placebo (n = 21)	Mean ± SD Oleoylethanolamide (n = 22)	P1	P2
FBS (mg/dL)				
Baseline	114.75 ± 5.16	116.04 ± 4.57	0.394	0.394
End	113.95 ± 5.43	101.681 ± 2.95	0.01	0.01
P3	0.401	0.01		
Mean changes	− 0.8 ± 0.27	− 14.35 ± 1.62	0.03	0.03
2hpp (mg/dL)				
Baseline	161 ± 9.14	162.50 ± 12.62	0.66	0.66
End	159.05 ± 9.88	136.68 ± 10.94	0.01	0.01
P3	0.52	0.01		
Mean changes	− 1.95 ± 0.73	− 25.82 ± 1.68	0.041	0.041
HbA_1_c (%)				
Baseline	6.340 ± 0.565	6.486 ± 0.535	0.394	0.394
End	6.250 ± 0.583	5.590 ± 0.361	0.01	0.01
P3	0.311	0.01		
Mean changes	− 0.09 ± 0.02	− 0.89 ± 0.17	0.02	0.02
Insulin (µU/ml)				
Baseline	12.37 ± 1.77	12.36 ± 1.73	0.378	0.378
End	12.2 ± 1.75	10.12 ± 1.11	0.01	0.01
P3	0.329	0.01		
Mean changes	− 0.17 ± 0.01	− 2.24 ± 0.62	0.031	0.031
HOMA-IR				
Baseline	3.51 ± 0.64	3.546 ± 0.587	0.269	0.269
End	3.44 ± 0.63	2.537 ± 0.287	0.01	0.01
P3	0.207	0.01		
Mean changes	− 0.07 ± 0.01	− 1.01 ± 0.3	0.038	0.038
CRP (µM)				
Baseline	7.99 ± 0.54	7.87 ± 0.52	0.46	0.46
End	7.91 ± 0.59	7.03 ± 0.68	0.03	0.03
P3	0.39	0.034		
Mean changes	− 0.08 ± 0.05	− 0.84 ± 0.16	0.02	0.02

Data are expressed as means ± SD

*FBS *fasting blood sugar, *2-hpp *2-hour post prandial, *HOMA-IR* homeostatic model assessment for insulin resistance, *HbA*_1_*c* hemoglobin A_1_c, *CRP* C-reactive protein

P1: Comparison the mean of glycemic status and inflammatory factor between the two groups of OEA and placebo (Independent samples t-test)

P2: Comparison the mean of glycemic status and inflammatory factor between the two groups of OEA and placebo were resulted from ANCOVA in the adjusted models (adjusted for BMI, Physical activity and Metformin)

P3: Comparison of mean of glycemic status and inflammatory factor in each group at baseline and end of study (Paired samples t- test)

## Discussion

Today, prediabetes is on the rise along with diabetes [20]. Controlling blood sugar has reduced mortality and increased life expectancy, but there are still many patients who suffer from long-term complications of the disease, so, preventing pre-diabetes to diabetes is more important to prevent chronic complications [21]. Recent studies have shown that IR, oxidative stress, and inflammation worsen a patient’s glycemic status [5]. On the other hand, receiving dietary foods and supplements with antioxidant potential, by increasing insulin sensitivity, improving the state of oxidative stress to antioxidants and reducing inflammation, causes better control of blood sugar [2]. One of the dietary supplements is OEA fatty acid, whose anti-inflammatory and antioxidant properties have been reported in various scientific studies [16]. The aim of this study was to evaluate the consumption of 125 mg of OEA on some biochemical factors such as FBG, 2hpp, HbA_1_c, IR and CRP in pre-diabetic individuals. After eight weeks of supplementation, the results of the study showed that the use of 125 mg of OEA significantly reduced FBG, 2hpp and HbA_1_c in people with prediabetes. Also, fasting insulin level and HOMA index at the end of the study in the intervention group compared to the placebo group had a significant decrease. According to a search of a scientific database, a clinical trial report has not been published to evaluate the effects of OEA in pre-diabetic individuals.

A clinical trial conducted in 2020 by Tutunchi et al. to investigate the effect of OEA supplementation on metabolic factors and appetite-related enzymes in obese people with fatty liver [19]. In their study, participants in the intervention group received daily OEA supplement for 12 weeks. At the end of the study, supplementation with OEA significantly reduced FBG, insulin and IR levels. However, the changes at the end of the study compared to the beginning of the study was not significant for HBA_1_c factor. The results of Tong Ren et al., study showed that receiving OEA reduced hyperglycemia in mice. In their study, doses of 15, 30 and 60 mg/body weight were given to mice for 56 days. Analysis of the study results showed that OEA increased glucose metabolism and decreased glucose concentration after 8 h of exposure. Serum insulin levels and IR also decreased in dose-dependent conditions [22].

Contrary to the mentioned studies, several animal investigations have not reported a significant effect of acute or chronic OEA intake on glucose levels [23, 24]. Impaired glucose metabolism and no change in serum insulin levels after acute treatment with 5 mg OEA / kg body weight have been reported in an animal study [25]. The difference between the results of scientific studies may be related to the different doses used in OEA, the duration of administration or the type of administration, whether acute or chronic. The mechanisms of action of OEA on metabolic factors, including glycemic index, are not fully understood due to the lack of sufficient reports from studies in different cellular, animal and human categories. Several studies have been performed on animals who Peroxisome proliferator-activated receptor alpha (PPAR-α) - knockout, is suggesting a specific role for PPAR-α in the metabolic effects of OEA [26]. Therefore, a possible reason for the improvement of glycemic status after receiving this fatty acid may be partly due to the expression of the PPAR-α gene. According to scientific reports, PPAR-α activation regulates glucose homeostasis metabolism by increasing insulin sensitivity in adipose and muscle tissue. Also, the role of this receptor in regulating the expression of several genes controlling β-cell function has been shown in scientific studies [27, 28]. Major expression of the G protein-coupled receptor 119 (GPR119) gene occurs in intestinal L cells and pancreatic β cells [29]. Binding of OEA to this receptor enhances the effect of GPR119 agonist on the secretion of glucagon-like peptide (GLP-1) [29]. The role and importance of GLP-1, as a potent hormone in regulating glucose metabolism has been known for many years. This incretin hormone increases insulin sensitivity and glucose uptake into adipose and muscle tissue in living organisms. Also, an increase in direct glucose excretion and finally a decrease in IR by this hormone has been reported [30]. Considering the possible mechanisms mentioned, the improvement of glycemic status after receiving OEA in people with prediabetes with GLP-1 secretion may be justified.

Also in the present study, supplementation with OEA fatty acid significantly reduced the inflammatory factor CRP at the end of the study. In a study by Payahoo et al. the effect of OEA on some inflammatory factors in obese individuals was investigated. Their double-blind study was performed on 60 obese individuals. Subjects were divided into intervention and control groups and the intervention group received OEA daily for 8 weeks. The final results of their study indicated that consumption of OEA caused a significant decrease in IL6 and TNFα levels [16]. Various scientific investigations show that inflammatory factors play an important role in creating and increasing IR [5]. Increased CRP concentrations have been reported in people with prediabetes [31]. In a case-control study conducted by Mahat, Roshan Kumar et al., on 400 individuals, the data showed that CRP levels in the prediabetes group were significantly higher than in the control group [32]. Based on the results of studies has shown a positive relationship between this inflammatory factor and glycemic disorder. These findings suggest that chronic inflammation may be a trigger for the development of type 2 diabetes [4]. Increasing the concentration of CRP in prediabetes may reduce insulin sensitivity and eventually worsen glycemic status by raising blood sugar. On the other hand, inflammation and oxidative stress are bilaterally related [2]. Increased inflammatory factors further upset the balance between the antioxidant system and oxidants, and exacerbate oxidative stress [9]. The findings of clinical studies indicate the anti-inflammatory and antioxidant properties of OEA. Intake of OEA fatty acids can increase IL10 levels as an anti-inflammatory cytokine. OEA exhibits its antioxidant and anti-inflammatory effects in a variety of ways. OEA fatty acid binds to PPAR-α and reduces the production of ROS and proinflammatory cytokines [14, 23]. Also, this fatty acid increases the activity of antioxidant enzymes and reduces fat peroxidation by protecting cells and cellular receptors, causing better insulin function and reducing IR.

This clinical trial, like other clinical studies, has strengths and weaknesses. One of the strengths of this study was that for the first time the effect of pure OEA supplementation in pre-diabetic patients on glycemic status and IR was investigated. On the other hand, designing this study as a double-blind randomized clinical trial with parallel groups, the results of this study are considered. Control of confounding factors such as weight, physical activity and food intake is also important in studies on people with metabolic diseases, which has been done in this study. However, due to the low budget and limited number of participants and the short duration of the intervention, the results of this study have been statistically analyzed. It should be noted that for clinical conclusions and better evaluation of clinical effects, it is necessary. Studies should be done with the number of people, longer duration and different doses of supplements.

## Conclusions

The results of this study showed that 8 weeks of supplementation with oleoylethanolamide at a dose of 125 mg per day can statistically improve glycemic status and inflammatory factor in patients with prediabetes. These results provide evidence to support the view that intake of this fatty acid or put its resources in the diet may play an important role in helping to control pre-diabetes status and prevent the shift to type 2 diabetes. However, further studies are needed to provide additional and convincing evidence.

## Data Availability

The datasets used and/or analyzed during the current study are available from the corresponding author upon reasonable request.

## Abbreviations

ADA: American diabetes association
BMI: Body mass index
BS: Blood sugar
CRP: C-reactive protein
FBG: Fasting blood glucose
GLP-: Glucagon-like peptide
GPR119: G protein-coupled receptor 119
HbA1c: Hemoglobin A_1_c
IFG: Impaired fasting glucose
IGT: Impaired glucose tolerance
IPAQ: International physical activity questionnaire
IR: Insulin resistance
OEA: Oleoylethanolamide
OGTT: Oral glucose tolerance test
OS: Oxidative stress
PPAR-α: Peroxisome proliferator-activated receptor alpha
ROS: Reactive oxygen species
2hpp: 2-hour Post Prandial
